# Factors Affecting Willingness on Sharing of Electronic Health Records Data: A Survey on Chinese Residents

This article has been retracted.

**DOI:** 10.1155/2022/5280792

**Published:** 2022-07-11

**Authors:** Ying He, Qiu He, Lun Li, Weihong Wang, Wenting Zha, Qian Liu

**Affiliations:** ^1^School of Medicine, Hunan Normal University, Changsha, Hunan, China; ^2^Faculty of Humanities and Social Sciences, Dalian University of Technology, Dalian, Liaoning, China

## Abstract

**Background:**

China has been promoting sharing of Electronic Health Records (EHRs) data for several years. However, only a few studies have explored the views of Chinese residents on sharing personal health data, and the factors that affect sharing of EHRs have not been fully elucidated. This study sought to explore public attitudes toward sharing EHRs and the factors that affect sharing of personal health data among Chinese residents.

**Methods:**

A multi-stage stratified sampling design was adopted in this survey to select residents in Hunan province, resulting in 932 responses randomly. The investigation was carried out with the administration of a 19-item questionnaire. The measure includes items on demographics, willingness to share EHRs, experiences on EHRs, public acknowledgment of the benefits of sharing EHRs, and public awareness of potential risks of sharing EHRs.

**Results:**

The score of general willingness to share EHRs was 5.784 ± 2.031. Concerning the domain scores for the willingness, the willingness to share EHRs for research was 2.060 ± 0.942, whereas sharing anonymization EHRs for other nonmedical services was only 1.805 ± 0.877. Multiple linear regression showed that general willingness to share EHRs was related to job-related healthcare (*β* = 0.520), experiences on EHRs (*β* = 0.192), public awareness of potential risks of sharing EHRs (*β* = −0.130), and public acknowledgment of the benefits of sharing EHRs (*β* = 0.290).

**Conclusion:**

The willingness to share EHRs data with Chinese residents was not high. The willingness of Chinese residents towards data sharing in EHRs is influenced by several factors, primarily job-related to healthcare, experiences on EHRs, public acknowledgment of the benefits of sharing EHRs, and public awareness of potential risks of sharing EHRs. The results provide a basis for related research and provide information for designing public health strategies such as formulating policies to improve public acceptance of sharing EHRs and promoting EHRs-based public health services.

## 1. Introduction

Advances in healthcare digitalization have improved the management of Electronic Medical Records (EMRs) and Electronic Health Records (EHRs), resulting in large clinical and health information data. Sharing these data through secure networks benefits multi-stakeholders, such as improving patient care, facilitating the allocation of medical resources, maintaining control of medical costs, and upgrading healthcare management. In the recent past, EHRs/EMRs have been transmitted from medical fields to a larger area covering social security systems and civil administrations, implying that sharing of these data improves the efficacy of public health authorities.

Public engagement is an essential part of an electronic health information exchange network. Over the past decade, there has been an increasing amount of literature on understanding the willingness, interest, and motivation to share health information. Sharing health information is nuanced by the influence of multiple factors, including personality traits, information privacy security, and other attributes related to the context around information sharing [1]. Details are discussed in four aspects as follows: (1) the demographic factors as a significant theme were primarily noted in the studies, including age, personal health conditions, social–economic status, and education levels. For example, It was reported that highly educated people had high confidence that sharing health data could improve public health and quality of care [2]. Other studies indicate nationalities [3], race [4], and personal computer experiences affect willingness to share personal health data [5–7]. (2) Data privacy was another important factor related to the willingness to share health information. The study showed that the concern of data privacy limited consent to sharing personal health data [8, 9]. In addition, previous IT experience was also associated with the willingness to share health information. Respondents who showed interest and engagement in IT were more accepting of sharing health records [10]. (3) Finally, the type and amount of health information associated with the willingness to share health information, especially the sensitive data, was the primary concern [11]. Overall, these studies indicated that a mix of sociodemographic factors, EHRs factors, and cognitive factors of health data influence willingness to share.

China has achieved a significant increase in EHRs/EMRs; however, the public view toward sharing EHRs/EMRs has not been fully explored. A better understanding of Chinese residents' views on sharing health data can facilitate healthcare management and enhance public trust in healthcare services. This study aims to explore the public view on sharing health data and the effect of factors. Our scientific contribution is twofold. First, this paper contributes to the literature on the public understanding of medical information technology. Our study focuses on public perceptions, understanding, and attitudes towards sharing transactional records for medical data linkage, which remains an under-explored area. Second, we quantify which demographic characteristics, privacy risks, and benefit expectations would most relevantly contribute to the willingness to share health data. To the best of our knowledge, few previous comprehensive researches have clarified these factors with China's public attitudes.

The remainder of the paper is arranged as follows: Section 2 describes the materials and methodology implemented in this study.  Section 3 provides the results of our empirical analyses.  Section 4 discusses the result that reflects the influence factors on willingness to share EHRs data and the substantive implications of our findings. Finally, Section 5 presents the conclusions that can be derived from this research.

## 2. Materials and Methods

### 2.1. Sampling Design

The sample size was calculated using the formula [12]:

(1) $$\begin{array}{c} N=deff\frac{\mu_{\partial }^{2}\times P\times \left(1-P\right)}{\zeta^{2}}, \end{array}$$

(*deff* *=* *1.5, u*_*α*_ = 1.96, *α* = 0.05, *δ* = 10% ^*∗*^ p). *P* is the support rate for sharing EHRs for different purposes (47.1% was considered the estimate for this sample size because it averaged between 38.9% and 55.2% in a previous study [13]). The sample size was calculated as 718. The minimum survey sample size was 862 considering 20% of the participants dropped out during the study.

Multistage stratified sampling method was used to randomly select participants from the residents of Hunan Province, China. The questionnaire designed in this study was distributed for the selection of residents from April 2019 to June 2019. The survey was approved by the Human Ethics Committee of Hunan Normal University (2019–204).

Cities and counties in Hunan Province were assigned into three categories based on their economic development levels reported in the Hunan Statistic Year Book 2012 [14]as follows: (1) The developed region where the GDP per capita was more than 85,000 RMB, including Chang-Zhu-Tan region; (2) The developing region where the GDP per capita was between 50,000 and 85,000 RMB, including six cities and their counties namely; Hengyang, Chenzhou, Yueyang, Loudi, Yiyang, and Changde; (3) The underdeveloped region where the GDP per capita was less than 50,000 RMB, including five cities and their counties, namely, Shaoyang, Yongzhou, Huaihua, Zhangjiajie, and Xiangxi Autonomous Prefecture. One city was randomly selected from each of the three categories and a resident committee that belongs to an urban area and a village that belongs to a county were further randomly selected from each of the three selected cities. Therefore, six basic strata were obtained from both geographically and economically different regions. Further, a minimum of 148 households were selected from each of the six strata, and one resident was randomly selected from each family as the survey respondent. The final survey sample size included 940 individuals, and the number of valid questionnaires obtained was 932, which was more than the required sample size.

### 2.2. Survey Domains and Instrument

The following measures were administered as part of a larger battery of questionnaires. Additional correlative studies will be described in other separate reports. The survey was designed following themes reported in previous literature [15], focus group discussions of the views, and influential factors reported previously. The core of the questionnaire was a set of 19 questions evaluating the willingness and influential factors on EHRs data sharing. General willingness to share EHRs was defined as the outcome variable, measured by 3 questions put on Likert's scale with three-point scales (1 = Disagree, 2 = Not sure, 3 = Agree). The score of general willingness to share EHRs was calculated based on the sum of the item scores, which ranged from 3 to 9. We categorized mean scores of > 3 to ≤ 4 as “low level of willingness,” > 4 to ≤ 7 as “moderate level of willingness,” and > 7 to ≤ 9 as “high level of willingness.” Three explanatory variables were defined using a five-point answering scale with the extremes labeled as “poor” and “excellent,” including experiences on EHRs (4 questions), public acknowledgment of the benefits of sharing EHRs(2 questions), public awareness of potential risks of sharing EHRs (4 questions). Meanwhile, participants recorded their demographic data on the questionnaires (6 questions). The questionnaires were distributed to 30 people of different ages, genders, education levels, health conditions, and healthcare experiences for a pilot study. The questionnaire was revised based on the responses of the 30 subjects.

After the whole survey had closed, we calculated the reliability scores for the scales in the study. The reliability questionnaire consisted of those questions from the original questionnaire most relevant to the central study hypothesis, with no demographic information. The findings indicated that the questionnaire had good reliability, with a Cronbach's *α* of 0.713.

The questionnaire was deployed using an online survey platform called Wen Juan Xing (WJX) and was sent to participants through e-mail and WeChat (a social media APP).

### 2.3. Statistical Analysis

Statistical Analysis Data were analyzed by SPSSAU (https://spssau.com/), a software package that comes with WJX, which has similar statistical algorithms used in SPSS. Continuous variables were expressed as mean ± standard deviation, whereas frequencies were calculated for categorical variables. Statistical analysis included Kolmogorov–Smirnov test for normality, nonparametric tests (Kruskal-Wallis test and Mann–Whitney *U* test), and Spearman correlation analysis. Multiple stepwise regression analysis was conducted to explore the factors influencing willingness to share EHRs. A *p* value of 0.05 for a covariate in the final model was considered statistically significant.

## 3. Results

### 3.1. Sample Characteristics

Out of the 932 respondents, 649 (71%) were aged between 18 and 45 years; 393 (42.58%) were male, and 530 (57.42%) were female. Approximately half of the participants (414, 44.85%) had completed a college education, and about half of the participants (414, 44.85%) were from families with a household income between 2,000 and 5,000 RMB per month. The results showed that 199 (21.56%) respondents worked at public institutions, whereas 193 (20.7%) participants were freelancers.

### 3.2. Willingness to Share EHRs

The score of general willingness to share EHRs ranged from 3 to 9, with a mean score of 5.784 and a standard deviation of 2.031. More than half of the sample (464, 50.27%) had negative attitudes toward the willingness to share EHRs, which scored less than the mean score of 5.7. In detail, only 22.1% (*n* = 247)of people scored high (8–9), while 51.14% (*n* = 472) and 26.76% (*n* = 204) scored medium (5–7) and low (3–4), respectively.

Concerning the domain scores for the willingness, the willingness to share EHRs for research (2.060 ± 0.942) yielded the highest average score. In contrast, the score of share anonymisation EHRs for other nonmedical services (1.805 ± 0.877) was the lowest. The individual and total scores for willingness to share were presented in Table 1.

### 3.3. Comparison of General Willingness to Share EHRs Based on Different Demographic Variables

The Kolmogorov-Smirnov test for normality showed that the distribution of general willingness to share EHRs was significantly different than normal (*D* = 0.153, *p* < 0.001). The data were nonnormally distributed. Therefore, nonparametric testing Kruskal–Wallis and Mann–Whitney U were used for difference and associations between the demographic variables with general willingness to share EHRs. A statistically significant interaction was found for age and job-related to healthcare. The results are exhibited in Table 2 and Figure 1.

### 3.4. The Correlation Analysis between General Willingness to Share EHRs and Experiences on EHRs, Public Awareness of Potential risks, and Public Acknowledgment of the Benefits

To analyze the correlation between general willingness to share EHRs and experiences on EHRs, public awareness of potential risks, and public acknowledgment of the benefits; the Pearson correlation analysis with scatter plots (Figure 2) was used. Corresponding results revealed that experiences with EHRs(*r* = 0.280, *p* < 0.001), and public acknowledgment of the benefits of sharing EHRs(*r* = 0.253, *p* < 0.001)were positively correlated with general willingness to share EHRs. Meanwhile, there were negative correlations of general willingness to share EHRs and public awareness of potential risks of sharing EHRs (*r* = −0.125, *p* < 0.001).

### 3.5. Multiple Stepwise Regression Analysis of General Willingness to Share EHRs

Multiple stepwise regression analysis (*α*_in_ = 0.05, *α*_out_ = 0.10) was performed to explore further the factors associated with general willingness to share EHRs and identify its independent determinants. General willingness to share EHRs was defined as the dependent variable and age (<18 = 1, 18–45 = 2, 45–60 = 3, > 60 = 4), job-related to healthcare (No = 0, Yes = 1), experiences on EHRs, public awareness of potential risks of sharing EHRs, and public acknowledgment of the benefits of sharing EHRs entered into the model as independent variables.

The prediction models established by stepwise regression were shown in Table 3 and Figure 3. The only independent variable not entered into the multivariable model was age. The results indicated that people who presented the following characteristics were more likely to consent to share EHRs: (1) worked in a healthcare-related position; (2) Having experiences with EHRs; (3) those who valued the potential benefits of sharing EHRs; (4) those who disagreed potential risks of sharing EHRs (*p* < 0.001; Figure 3).

## 4. Discussion

### 4.1. General Willingness to Share EHRs

The present study explored factors associated with EHRs data sharing among residents in China. The total score of general willingness ranged from 3 to 9. However, the mean score of 5.784 ± 2.031 meant a moderate level. Moreover, the score of share anonymisation EHRs for other nonmedical services was only 1.805 ± 0.877. Thus, the willingness to share EHRs data with Chinese residents was not high. This finding is consistent with a previous study reported in China whereby only 38.9% of the public would like to use their EHRs for medical research, 30% for other nonmedical services [11]. This result is comparable to the rate in other countries, including California (56.4%) [13], but slightly lower relative to the rate reported in the United Kingdom (62.47%) [16]. The study sought to determine that most Chinese residents held reservations about sharing EHRs.

The above results seem to be inconsistent with previous China's privacy culture results framework. Previous studies report that Chinese cultural history is a culture of shame based on Chinese traditional culture [17]. Cultural ideals of saint personality result in insufficient resources owing to the right to privacy. A study published in 2011 reported that China, India, and Brazil, had the highest percentage of users who frequently shared personal information online for their benefit [18].

However, the influence of traditional Chinese culture on the concept of privacy in contemporary China has decreased, owing to the significant changes in economy, culture, and social structure, and the recent popularity of the Internet. Digital information privacy is becoming increasingly important to Chinese residents. For example, a survey conducted by the China Youth Social Center indicated that most respondents (88.8%) had experienced improper processing of their data [19]. The findings of the present study show the consequences of mobile Internet and Big Data in the past few years, which reshapes Chinese' conceptualization of privacy which was not reported in McDougall's survey [18]. The results of the present study indicated that Chinese residents significantly associate privacy with their personal information, especially personal health data. The finding indicated an increase in the awareness of information privacy protection of Chinese residents.

### 4.2. Factors Affecting Willingness

The results of the study showed that the most influential factor of public preference for sharing data was the balance consideration between privacy protection and benefits for society. Respondents in the present survey, who agreed that sharing EHRs would benefit healthcare services and related research, were more likely to consent to share their data. Previous studies reported similar findings that the privacy and security of EHRs is an essential consideration for the public in deciding whether to share health information [1, 7, 20]. For instance, approximately two-thirds of American adults reported that the privacy of personal health data would be undermined during electronic transmission of the data [21]. A survey conducted based on 1,000 Americans demonstrated that 41.2% of the participants believed that sharing of EHRs would affect patients' privacy [2]. A previous study conducted among Greek participants reported that 48.8% of the participants were worried that an unauthorized third party would access their personal information [22].

Culnan and Armstrong's theory on privacy computing can explain these findings. The theory indicates that users who disclose personal information in exchange for some economic or social benefit are assessed to ensure that their private information is not used illegally and that the individual is not adversely affected [23]. Therefore, users are willing to reveal personal information in a transactional environment if the benefits outweigh the risks. People are more likely to expect some form of social gain from sharing their health information if the likelihood of privacy risk is low, or when the risks have a significant impact on specific individuals rather than most of the general population. For example, the public focus would incline to expected benefits or social gains of sharing EHRs when potential security threats are few or when they only target specific persons instead of most individuals in the population. This empirical survey further established that the balance consideration between privacy protection and benefits for society significantly influences the utilization of EHRs data. Further research should be conducted to reduce the propaganda that affects EHRs sharing, come up with utilization policies, increase the protection of personal privacy, and reduce the public's concern about privacy leakage of individual EHRs data.

Some findings in the current study reflect the Chinese cultural and policy context, which is different from the findings reported in Western developed countries. Four demographic characteristics were included in the questionnaire, but the results showed that only one demographic factor was associated with a general willingness to share health data namely whether the participant's job is related to healthcare.

One notable finding was that young respondents (5.653 ± 2.026) are less likely to have positive views of EHRs than older respondents (6.257 ± 2.254). This finding is a contrast to other studies. For example, a survey conducted in the UK reported that younger participants (25–34 years old) were more likely to support sharing of EHRs information compared with older participants (35–64 years old) [24]. It seemed that the relationship between age and willingness to share health information was contested. Some studies reported that older people were more willing to share health information because of a higher level of involvement with the health care system [25]. In contrast, other studies found older people had less willing to share, as they were less comfortable with information technology, especially sharing health information via mobile phone apps [26]. These differences suggested that the exploration of the age to share health information may be incomplete. We speculated that there could be three possible reasons. Firstly, age may work together with other sociodemographic factors to influence the willingness. Therefore, future studies would need to analyze different sociodemographic factors and stratify them to rule out possible confounding. Secondly, most demographic characteristics were related to local cultures, beliefs, and conditions of sharing EHRs, thus could explain the variations among countries in part. Additionally, this may be related to the sample size difference because the number of elderly individuals (35,3.39%) was small among our samples. The sample size needed to be expanded for more in-depth research in the future.

Further, participants who had their EHRs experiences were more willing to give consent for sharing of EHRs. This might be because consumers who had used EHRs may have helped these participants to better understand EHRs and gain immediate impressions of perceived benefits and risks. China has made significant progress in the generation and utilization of medical big data in recent years. The national rate of EHRs for residents was 76.4% by the end of 2015 [27]. This finding indicates that expanding EHRs users would promote EHRs and further improve sharing of EHRs. These findings provide empirical evidence for the replication of data sharing for EHRs in other countries.

### 4.3. Limitations of the Study

The study was a single-site study limited within Hunan Province, China. Therefore, findings related to demographic characteristics may not be generalized to other populations. The multi-stage stratified sampling used in the present study eliminated bias as much as possible; however, the resulting samples roughly shared a similar profile as follows: young, highly educated, and sensitive to privacy. Further studies with larger sample sizes and comprising different groups should be conducted to verify the findings.

The questionnaire used in the current study focused on general attitudes toward EHRs, instead of explaining specific scenarios. Therefore, interpretations of the questions, especially questions related to privacy and security, varied among participants and subsequently affected the answers provided. Descriptions of practical projects or real-life situations should be included in further studies.

## 5. Conclusion

Most residents in Hunan Province are cautious about sharing EHR data. Notably, the reticence level was on topics of EHRs sharing between different institutions or for use beyond healthcare scope was significantly high. Factors that affect general willingness to sharing of EHR data include jobs related to healthcare, having EHRs experiences, and awareness of benefits and risks of sharing EHRs [28].

The findings of the present study reveal important factors for improving healthcare services in multi-aspects. Responses to the questionnaire indicated why people hesitate to share EHRs data. These reasons can provide a basis for administrators to develop specific strategies targeting public acceptance of storing and sharing of EHRs, improve public confidence in sharing EHRs, and lay a basis for further studies on extensive medical data. Further studies should explore related issues such as the scope and types of personal health data to be shared, forms of informed consent for allowing sharing of health data, identification of personal health characteristics, and measures for privacy protection.

## Figures and Tables

**Figure 1:** Boxplots of statistical results: (a) age; (b) job related to healthcare.

**Figure 2:** Scatterplot analysis of the correlation between general willingness to share EHRs with (a)experiences with EHRs; (b)public acknowledgment of the benefits of sharing EHRs; (c) public awareness of potential risks of sharing EHRs.

**Figure 3:** Linear regression model of Independent factors related to willingness to share EHRs.

**Table 1:** Individual and total willingness to Share EHRs scores.

	Mean ± SD
General willingness to share EHRs	5.784 ± 2.031
Willingness to share anonymisation EHRs for research	2.148 ± 0.884
Willingness to share anonymisation EHRs for other nonmedical services	1.805 ± 0.877
Willingness to share anonymisation EHRs between different institutions	1.831 ± 0.886

**Table 2:** Comparison of willingness to share EHRs based on different demographic variables.

Characteristics	*x* ± *s*	*Z/H* ^*∗*^	*p*
Age			
<18	6.111 ± 2.082	9.894	0.019
18–45	5.653 ± 2.026		
45–60	6.066 ± 1.968		
>60	6.257 ± 2.254		

Job-related to healthcare			
Yes	6.322 ± 1.977	−3.832	0.001
No	5.660 ± 2.024		

*p* < 0.01. ^*∗*^Mann–Whitney test was used for statistical analysis of two groups and *Kruskal–Wallis* test for more than two groups.

**Table 3:** Multi-variable linear stepwise regression results.

	*B*	*SE*	*Beta*	*95% CI*	*T*	*p*
Constant	3.987	0.400	—	3.203 ∼ 4.771	9.968	0.001^*∗∗*^
Job-related to healthcare	0.520	0.158	0.100	0.209 ∼ 0.831	3.282	0.001^*∗∗*^
Experiences on EHRs	0.192	0.030	0.203	0.133 ∼ 0.251	6.352	0.001^*∗∗*^
Public awareness of the potential risks of sharing EHRs	−0.130	0.020	−0.203	−0.169 ∼ −0.090	−6.440	0.001^*∗∗*^
Public acknowledgment of the benefits of sharing EHRs	0.290	0.039	0.245	0.214 ∼ 0.367	7.439	0.001^*∗∗*^

^*∗∗*^ *p* < 0.001. *R*^*2*^ = 0.159, *F* (4,918) = 43.331, *p* < 0.001.

## Data Availability

The datasets used or analyzed in the current study are available from the corresponding author on reasonable request.

## Abbreviations

EHRs: Electronic health records
EMRs: Electronic medical records.

## References

[1] Weitzman E. R., Kelemen S., Kaci L., Mandl K. D. (2012). Willingness to share personal health record data for care improvement and public health: a survey of experienced personal health record users. *BMC Medical Informatics and Decision Making*.

[2] Ancker J. S., Brenner S., Richardson Joshua E., Silver M., Rainu K. (2015). Trends in public perceptions of electronic health records during early years of meaningful use. *American Journal of Managed Care*.

[3] Grande D., Mitra N., Shah A., Wan F., Asch D. A. (2013). Public preferences about secondary uses of electronic health information. *JAMA Internal Medicine*.

[4] Dimitropoulos L., Patel V., Scheffler S. A., Posnack S. (2011). Public attitudes toward health information exchange: perceived benefits and concerns. *American Journal of Managed Care*.

[5] Luchenski S. A., Reed J. E., Marston C., Papoutsi C., Majeed A., Bell D. (2013). Patient and public views on electronic health records and their uses in the United Kingdom: cross-sectional survey. *Journal of Medical Internet Research*.

[6] Luchenski S., Balasanthiran A., Marston C. (2012). Survey of patient and public perceptions of electronic health records for healthcare, policy and research: study protocol. *BMC Medical Informatics and Decision Making*.

[7] Buckley B. S., Murphy A. W., MacFarlane A. E. (2011). Public attitudes to the use in research of personal health information from general practitioners’ records: a survey of the Irish general public. *Journal of Medical Ethics*.

[8] Weitzman E. R., Kaci L., Mandl K. D. (2010). Sharing medical data for health research: the early personal health record experience. *Journal of Medical Internet Research*.

[9] Caine K., Hanania R. (2013). Patients want granular privacy control over health information in electronic medical records. *Journal of the American Medical Informatics Association*.

[10] Cocosila M., Archer N. (2014 23). Perceptions of chronically ill and healthy consumers about electronic personal health records: a comparative empirical investigation. *BMJ Open*.

[11] Pedersen H., Taylor D., Gilbert M., Achen M., Lester R., Ogilvie G. (2015). A cross-sectional survey exploring attitudes towards provincial electronic health record implementation among clients attending the provincial sexually transmitted infections clinic in British Columbia. *Sexually Transmitted Infections*.

[12] Hu J., Jiang W., Lin X. (2018). Dental caries status and caries risk factors in students ages 12–14 Years in zhejiang, China. *Medical Science Monitor*.

[13] Zhong Q. (2019). Investigation and analysis of privacy protection for electronic health records in China-from the perspective of the public. *Archival Research*.

[14] (2012). *Hunan Statistical Bureau, Hunan Statistic Yearbook*.

[15] Kim K. K., Sankar P., Wilson M. D., Haynes S. C (2017). Factors affecting willingness to share electronic health data among California consumers. *BMC Medical Ethics*.

[16] Luchenski S. A., Reed J. E., Marston C., Papoutsi C., Majeed A., Bell D (2013). Patient and public views on electronic health records and their uses in the United Kingdom: cross-sectional survey. *Journal of Medical Internet Research*.

[17] Chang L. (2003). A review of the study of public and private concepts in China[J]. *Nankai Journal*.

[18] Dutta S., Dutton W. H., Law G. (2011). The new Internet world: a global perspective on freedom of expression, privacy, trust and security online. *INSEAD Working Papers Collection*.

[19] Entzeridou E., Markopoulou E., Mollaki V. (2018). Public and physician’s expectations and ethical concerns about electronic health record: benefits outweigh risks except for information security. *International Journal of Medical Informatics*.

[20] Agaku I. T., Adisa A. O., Ayo-Yusuf O. A., Connolly G. N (2014). Concern about security and privacy, and perceived control over collection and use of health information are related to withholding of health information from healthcare providers. *Journal of the American Medical Informatics Association*.

[21] Ancker J. S., Silver M., Miller M. C., Kaushal R. (2013). Consumer experience with and attitudes toward health information technology: a nationwide survey. *Journal of the American Medical Informatics Association*.

[22] Senteio C., Veinot T., Adler-Milstein J., Richardson C (2018). Physicians’ perceptions of the impact of the EHR on the collection and retrieval of psychosocial information in outpatient diabetes care. *International Journal of Medical Informatics*.

[23] Culnan M. J., Armstrong P. K. (1999). Information privacy concerns, procedural fairness, and impersonal trust: an empirical investigation. *Organization Science*.

[24] Healthcare Foundation National consumer health privacy survey 2005. https://www.chcf.org/publications/2005/11/national-consumer-health-privacy-survey-2005.

[25] Brown S. M., Bell S. K., Roche S. D. (2016). Preferences of current and potential patients and family members regarding implementation of electronic communication portals in intensive care units. *Annals ATS*.

[26] Cocosila M., Archer N. (2014). Perceptions of chronically ill and healthy consumers about electronic personal health records: a comparative empirical investigation. *BMJ Open*.

[27] National Health Planning Commission National electronic health records of residents reach 76.4% [eb/ol]. (2021-09-09). https://www.cankaoxiaoxi.com/china/20170710.

[28] Ying H., Lun L., Weihong W. Factors affecting views on electronic health data sharing:a survey of chinese residents. https://assets.researchsquare.com/files/rs-727836/v1/5c8c35a9-ddc9-417d-9090-b10acb6c07a2.pdf?c=1635344060.

